# miRNA-144-5p/ITGA3 Suppressed the Tumor-Promoting Behaviors of Thyroid Cancer Cells by Downregulating ITGA3

**DOI:** 10.1155/2021/9181941

**Published:** 2021-12-13

**Authors:** Jizong Zhang, Yan Zhong, Yiming Sang, Guanghui Ren

**Affiliations:** Department of Nail and Breast Surgery, Nanjing Second Hospital, 210009, Nanjing, Jiangsu Province, China

## Abstract

**Objective:**

To ascertain the mechanism of miRNA-144-5p and ITGA3 in thyroid cancer (TC).

**Methods:**

From The Cancer Genome Atlas (TCGA), RNA expression profiles were obtained for the expression analysis of miRNAs and mRNAs in TC. qRT-PCR and western blot were utilized to measure the expression of miRNA-144-5p and ITGA3 at RNA and protein levels, respectively. The association between miRNA-144-5p and ITGA3 was validated by the dual-luciferase assay. CCK-8, scratch healing, transwell, and flow cytometry assays were employed to evaluate tumor-related cell behaviors.

**Results:**

Low-expressed miRNA-144-5p and high-expressed ITGA3 were found in TC cells relative to normal cells. miRNA-144-5p expression was positively associated with suppressive effects on proliferative, invasive, and migratory ability of TC cells while negatively associated with cell apoptosis. miRNA-144-5p inhibited ITGA3 expression in TC, and its overexpression remarkably reversed the tumor-promoting effects of overexpressed ITGA3 on the biological functions of TC.

**Conclusion:**

It is verified in our study that cell growth of TC is inhibited by the miRNA-144-5p/ITGA3 axis, which represents an underlying target for TC. This research proposed a new insight into the strategy of TC treatment.

## 1. Introduction

Thyroid cancer (TC) is considered endocrine cancer, with continuous increasing morbidity in the past decades [1]. TC could be classified into different subtypes, where papillary thyroid cancer (PTC) occupies the majority of the new TC cases [2]. Treated with specific methods such as surgery, radioiodine, and thyroid-stimulating hormone suppression, a great number of patients showed a relatively optimal improvement in their condition. However, there was still recurrence and metastasis of the tumor [3–5]. Also, due to the unmatured prognostic assessment for TC patients, many patients suffered the overtreatment [6]. Considering the challenges of TC therapy and prognosis, it is of significance to carry out an in-depth exploration into the molecular mechanisms of TC, which is able to provide valuable insights into the developments of therapy and prognostic assessment.

Dysregulation of miRNAs was indicated by many studies to be heavily associated with tumor process [7]. Also, miRNAs are regarded as novel cancer biomarkers [8–10]. Among many miRNAs dysregulated in many cancer, miRNA-145 was reported as the tumor suppressor of cervical cancer [11], lung adenocarcinoma [12], and gastric cancer [13]. By bioinformatics analysis, miRNA-144-5p is lowly expressed in TC and implicated with cell adhesion and cell migration [14]. But experimental data are lacking, within a need of experiments to validate the possible impact of miRNA-144-5p on TC progression.

Integrin *α*3 (ITGA3), a cell surface adhesion molecule, is mainly expressed in the cell membrane. It was reported that ITGA3 can interact with extracellular matrix protein, and its expression is associated with cancer metastasis [15]. Besides, research on the molecular mechanism, results of bioinformatics analysis showed that ITGA3 is regarded as a pivotal biomarker for pancreatic cancer and can facilitate cancer progression through P53/TGF-*β*-related pathways [16]. Upregulation of ITGA3 exerts a promotive role in the cell proliferation of intrahepatic cholangiocarcinoma and indicates a poor prognosis [17]. Although some mechanisms of ITGA3 in TC were reported [18], the detailed functions and potential mechanisms of ITGA3 in TC are still unknown. Therefore, the study of the regulatory effect of ITGA3 on TC can improve the theoretical construction of ITGA3 as a cancer regulator.

To sum up, the current study focused on the effects of miRNA-144-5p and ITGA3 on TC, and miRNA-144-5p/ITGA3 regulatory axis was determined by bioinformatics methods and dual-luciferase assay. The findings in this study provided a new theoretical support for TC therapy.

## 2. Materials and Methods

### 2.1. Bioinformatics Methods

From The Cancer Genome Atlas (TCGA) (https://portal.gdc.cancer.gov/), mature miRNA (normal: 59, tumor: 514), mRNA expression data (normal: 58, tumor: 510), and clinical data (December 19, 2019) of TC were obtained. Then, differentially expressed miRNAs (DEmiRNAs) and mRNAs (DEmRNAs) were accessed by differential analysis (∣logFC | >1.5, *p*adj < 0.05). The prediction of the target miRNA was conducted through miRTarBase (http://mirtarbase.mTC.nctu.edu.tw/php/index.php) and TargetScan (http://www.targetscan.org/vert_72/) databases to gain the DEmRNAs that had binding sites of the miRNA. Pearson correlation analysis was carried out on miRNA-144-5p and the candidate mRNAs to ascertain the target. Clinical staging analysis of target mRNA was conducted.

### 2.2. Cell Lines and Culture

Human normal thyroid cell line HTori-3 (BNCC338687), TC cell line TPC-1 (BNCC338689), FTC-133 (BNCC337959), KTC-1 (BNCC340144), and 8505C (BNCC340524) were procured from BeNa Culture Collection (China). F-12K medium (BNCC341829, BeNa, China) was prepared for culturing HTori-3, KTC-1 and 8505C, and RPMI-1640 medium (BNCC341471, BeNa, China) for FTC-133, and Leibovitz's L-15 (L-15) medium (BNCC341687, BeNa, China) for TPC-1. 10% fetal bovine serum (FBS) was contained in the above mediums where cell lines were incubated under standard culture conditions.

### 2.3. Cell Transfection

miRNA-144-5p mimics (miR-mimics), negative control mimics (miR-NC), pcDNA3.1-ITGA3 plasmid (oe-ITGA3) encoding ITGA3, and blank pcDNA3.1 plasmid (oe-NC) vectors were all procured from RiboBio (China). Complying with the operation instructions, Lipofectamine 2000 kit (Invitrogen, Carlsbad, USA) was in use to transfect mimics/plasmids into TC cell lines TPC-1 and FTC-133. Cells were used for further experiments 24 h after transfection.

### 2.4. Real-Time PCR

Trizol reagent (Life Technologies, USA) was used for extracting total RNA. The miScript II RT kit (Qiagen, USA) was used to revert miRNA and mRNA to cDNA. The miScript SYBR Green PCR Kit (Qiagen, Germany) was used to measure expression levels of miRNA and mRNA. Then, qRT-PCR was operated on Applied Biosystems® 7500 Real-Time PCR Systems (Thermo Fisher Scientific, MA). GAPDH was taken as the internal parameter for ITGA3, and U6 for miRNA-144-5p. Primer sequences are exhibited in Table 1. The 2^-*ΔΔ*Ct^ value was employed to assess the relative expression of miRNA-144-5p and ITGA3.

### 2.5. Western Blot Assay

Radio immunoprecipitation assay lysis buffer (Beyotime, China) was used to extract cell lysates. Quantified by the BCA protein assay kit (Beyotime, China), the proteins were separated by 12% SDS-PAGE and transferred onto the PVDF membrane. 5% skimmed milk powder was harnessed to keep the membrane sealed for 2 h; then, it was incubated overnight with primary antibodies at 4°C. Next, phosphate-buffered saline with Tween® was harnessed to rinse the membrane and it was cultured at room temperature with the secondary antibody for 2 h. Eventually, an enhanced chemiluminescence (ECL) kit (GE Healthcare, USA) was in use to detect protein signals. The primary antibodies rabbit anti-ITGA3 (ab131055, 0.3 *μ*g/ml) and rabbit anti-GAPDH (ab181602, 1 : 10,000) and secondary antibody goat anti-rabbit IgG (ab205718) were provided by Abcam (China).

### 2.6. Cell Counting Kit-8 (CCK8) Assay

96-well plates (2 × 10^4^ cells/well) were used here to inoculate and culture cells at 37°C with 5% CO_2_. Incubated for 0, 24, 48, 72, and 96 h, 10 *μ*l CCK-8 solution was supplemented (CK04; Dojindo Laboratories, Japan). After 2 h, the absorbance was assessed at 450 nm.

### 2.7. Transwell Assay

A 24-well transwell chamber (8 *μ*m aperture, BD Biosciences) was utilized in this assay for migratory ability and invasiveness of cancer cell detection. Coated with Matrigel, the upper chamber was filled with nearly 2 × 10^4^ cells. And a medium containing 10% FBS was added to the lower chamber. After 48 h, the invaded cells were fastened with methanol as well as stained with 0.1% crystal violet. Finally, they were photographed under an inverted microscope (DSX510i, Olympus, Japan).

### 2.8. Scratch Healing Assay

Six-well plates were employed here for cell inoculation. Upon the overall coverage of cells reached 80%, the monolayer of cells was gently scraped with the tip of a 200 *μ*l pipette. After 24 h, the wound areas of cells both in the transfection group and in the control group were measured. Those isolated cells were removed by twice washing with the culture solution. As for the regrowth of cells (24 h), a fresh medium was used. Finally, at 0 h and 24 h, the cell migration was observed and photographed.

### 2.9. Flow Cytometry

Transfected for 48 h, cells were collected and digested. Then, they were washed twice with PBS, resuspended in binding buffer, and then added with Annexin V-FITC and propidium iodide (PI). Finally, the cell apoptosis was tested by FACS Calibur flow cytometry (Becton Dickinson, CA, USA) and the data were analyzed.

### 2.10. Dual-Luciferase Assay

The pmirGLO luciferase reporter vectors (Promega, USA) inserted with the ITGA3 wild-type (ITGA3-WT) and mutant (ITGA3-MUT) 3′-UTR were constructed to identify the binding relationship of miRNA-144-5p to the 3′-UTR of ITGA3. TC cell line TPC-1 was seeded in triplicate in 96-well plates (3 × 10^5^ cells/well), and 100 nM miR-mimics/miR-NC and ITGA3-WT/ITGA3-MUT plasmids were cotransfected into the cells. Cultured for 48 h, the dual-luciferase reporter system (Promega, USA) was then used for measuring the luciferase activity.

### 2.11. Statistical Analysis

Analysis of data from 3 independent experiments was conducted on GraphPad Prism 6.0 (La Jolla, CA). The results are expressed as mean ± standard deviation. Comparison between the two groups was Student's *t*-test, and comparison between multiple groups was one-way analysis of variance used for pretest. Then, the Bonferroni method was used for posttest.

## 3. Results

### 3.1. The Expression of miRNA-144-5p Is Notably Decreased in TC Cells

miRNA-144-5p was pointed out by the previous study as a TC-related miRNA by bioinformatics analysis [14]. However, no practical supports determine its molecular mechanisms in TC. To determine its roles in TC, we introduced the experiments in the following. A total amount of 82 DEmiRNAs were screened via differential expression analysis, including miRNA-144-5p which was the focus of our research (Figure 1(a)). Bioinformatics analysis of TCGA TC data indicated that TC was implicated in low miRNA-144-5p expression (Figure 1(b)). miRNA-144-5p expression in TC cell lines was markedly low as manifested in the qRT-PCR result (Figure 1(c)). These findings indicated that miRNA-144-5p was significantly low-expressed in TC.

### 3.2. Suppressive Effects of miRNA-144-5p on the Development of TC Cell Lines *In Vitro*

miRNA-144-5p expression level in FTC-133 and TPC-1 cell lines was notably different from that in the normal cell line; hence, they were chosen for the following functional experiments. After successful transfection of miRNA-144-5p mimic and miR-NC (negative control), miRNA-144-5p expression levels were assessed by qRT-PCR. Remarkable overexpression of miRNA-144-5p was observed in these two thyroid cancer cells compared with stimulated transfected cancer cells (Figure 2(a)), indicating these cells could be used in the subsequent experiments. Proliferation of TC cells was dramatically suppressed by miRNA-144-5p overexpression (Figure 2(b)). The invasiveness and mobility of these two thyroid cancer cells after overexpressing miRNA-144-5p were remarkably downregulated (Figures 2(c) and 2(d)). The flow cytometry result suggested that overexpressing miRNA-144-5p notably upregulated the apoptosis level of TC cells (Figure 2(e)). Collectively, proliferative, migratory, and invasive TC cells could be weakened by overexpression of miRNA-144-5p, while activating apoptosis.

### 3.3. ITGA3 Was Negatively Correlated with miRNA-144-5p Expression in TC Cells

To explore the downstream targets of miRNA-144-5p in TC cells, differential expression analysis was conducted on mRNAs, where 1,749 DEmRNAs including 1,270 upregulated and 479 downregulated DEmRNAs were screened (Figure 3(a)). The target genes of miRNA-144-5p were predicted using miRTarBase and TargetScan databases. The 3 DEmRNAs sharing binding sites with miRNA-144-5p were obtained by intersecting the predicted targets and the upregulated DEmRNAs (Figure 3(b)). It was revealed by the Pearson correlation analysis that miRNA-144-5p was negatively correlated with ITGA3 with the highest correlation coefficient (Figure 3(c)). Data from TCGA database indicated that ITGA3 was markedly overexpressed in TC tissue (Figure 3(d)). Combined with clinical information, the expression of ITGA3 was markedly different in patients with different T stages (Figure 3(e)) and N stages (Figure 3(f)) of the tumor. mRNA expression of ITGA3 in TC cell lines was significantly higher compared with that in normal cell line (Figure 3(g)). Similarly, the result of the western blot assay demonstrated that the protein level of ITGA3 in TC cell lines was considerably higher in contrast with that in normal cell line (Figure 3(h)). Based on the above results, ITGA3 could be one target of miRNA-144-5p.

### 3.4. miRNA-144-5p Suppresses ITGA3 Expression by Targeting It

We bioinformatically predicted that on the 3′UTR of ITGA3 existed the binding site of miRNA-144-5p (Figure 4(a)). Afterward, the targeted interaction was determined by dual-luciferase assay, where the luciferase activity was reduced by introducing miR-mimics in the ITGA3-WT group, indicating that the miRNA-144-5p binding site predicted by bioinformatics analysis was correct (Figure 4(b)). It was revealed by the qRT-PCR that overexpressed miRNA-144-5p markedly downregulated ITGA3 mRNA level in TC cells (Figure 4(c)). The ITGA3 protein expression was also notably reduced upon the overexpressing of miRNA-144-5p (Figure 4(d)). It was shown that miRNA-144-5p both reduced the translation and accelerated the mRNA degradation of ITGA3. In a word, these results suggested that miRNA-144-5p downregulated ITGA3 by targeting its 3′UTR region in TC cells.

### 3.5. miRNA-144-5p Suppresses TC Progression by Targeting ITGA3

When both miRNA-144-5p and ITGA3 were overexpressed, ITGA3 was strikingly upregulated in the miR-NC+oe-ITGA3 group while it was subsequently restored, or even downregulated (Figures 5(a) and 5(b)). CCK-8 assay results revealed that overexpressed ITGA3 remarkably enhanced the proliferative ability of TC cells. However, this promotive effect could be attenuated by the simultaneous overexpression of miRNA-144-5p and ITGA3 (Figure 5(c)). It was uncovered that the invasiveness as well as mobility of TC cells was markedly promoted after ITGA3 was overexpressed. But they were hugely decreased resulting from the simultaneous overexpression of miRNA-144-5p and ITGA3, in contrast with that when ITGA3 was overexpressed alone (Figures 5(d) and 5(e)). The overexpression of ITGA3 could prominently inhibit the cell apoptosis of TC, while the simultaneous overexpression of miRNA-144-5p and ITGA3 could reduce this inhibitory effect (Figure 5(f)). Thus, miRNA-144-5p partially rescued the phenotype induced by ITGA3 in TPC-1 cells. Overall, ITGA3 is suggested by these results to be a functional target of miRNA-144-5p.

## 4. Discussion

The expression status and potential roles of miRNA-144-5p were analyzed previously. For example, Pan et al. [14] pointed out that low expression of 4 miRNAs in TC, including miRNA-144-5p, may affect tumorigenesis through key pathways. Furtherly, it was verified by our study that expression of miRNA-144-5p was markedly downregulated in TC tissue and cells. The tumor-suppressing role of miRNA-144-5p in cell proliferation, migration, and invasion in TC was for the first time revealed by the results, presenting a novelty of our study. According to Rosignolo et al.'s research, miRNA-144-5p could be applied to classify PTC combined with other miRNAs [19], showing a promising potential; however; in our study, we failed to verify miRNA-144-5p expression status and effects among TC subtypes. In conclusion, we expanded the understandings on miRNA-144-5p to some extent based on the previous studies.

This study demonstrated that ITGA3 was possible to be the downstream target of miRNA-144-5p. It was reported that ITGA3 is highly expressed in different cancer types [16, 17]. Moreover, highly expressed ITGA3 was proved to stimulate the proliferation and metastasis of tumor cells in former studies [20]. Liu et al. [18] revealed that the growth of TPC cells was able to be reduced by miRNA-524-5p targeting FOXE1 and ITGA3. However, the detailed functions of ITGA3 in TC are still incomplete. Through cell biology experiments, the expression of ITGA3 was verified to be upregulated in TC cells, and the overexpression of ITGA3 enhances the proliferative, migratory, and invasive ability while weakening cell apoptosis of TC cells. Additionally, dual-luciferase assay results further verified the binding relationship between ITGA3 and miRNA-144-5p. And it was also uncovered that miRNA-144-5p attenuated the proliferative, migratory, and invasive ability and promoted cell apoptosis by targeting ITGA3. These conclusions provided a molecular mechanism for the migration and invasion of TC, helping to develop new therapeutic methods for TC.

In conclusion, we demonstrated in this study that miRNA-144-5p inhibited the progression of TC cells. And that this effect was mediated, at least in part, by ITGA3. Although we have initially explored the role of miRNA-144-5p/ITGA3 in the TC cell phenotype, further elucidation of its downstream pathways in thyroid cancer is indispensable, which is crucial for the development of effective diagnosis and treatment of thyroid cancer.

## Figures and Tables

**Figure 1:** miRNA-144-5p is notably decreased in TC cells: (a) volcano map of DEmiRNAs in TC data set with red representing upregulation while green representing downregulation; (b) expression of miRNA-144-5p; (c) miRNA-144-5p expression in normal cell line HTori-3 and TC cell lines TPC-1, FTC-133, KTC-1, and 8505C detected by qRT-PCR; ∗ denotes *p* < 0.05.

**Figure 2:** Overexpressed miRNA-144-5p suppresses malignant behaviors of TC cells: (a) transfection efficiency of miRNA-144-5p in TPC-1 and FTC-133 cell lines tested by qRT-PCR; (b) cell proliferation in miR-NC and miR-mimic groups tested by CCK-8; (c) cell invasion in s groups tested by transwell assay (100x); (d) cell migration in groups tested by scratch healing assay (40x); (e) cell apoptosis in groups tested by flow cytometry; ∗ denotes *p* < 0.05.

**Figure 3:** ITGA3 is remarkably highly expressed in TC cells: (a) volcano map of DEmRNAs in TC data set, with red representing upregulation while green representing downregulation; (b) Venn plot of predicted target mRNAs of miRNA-144-5p and differentially upregulated mRNAs; (c) Pearson correlation analysis diagram of miRNA-144-5p and target mRNAs; (d) ITGA3 level in normal and tumor cells; (e) boxplot of ITGA3 expression in different T stages; (f) boxplot of ITGA3 expression in different N stages of TC; (g) ITGA3 mRNA level in normal cell line and TC cell lines; (h) ITGA3 protein level in normal cell line and TC cell lines; ∗ denotes *p* < 0.05.

**Figure 4:** miRNA-144-5p is the upstream regulator of ITGA3: (a) the binding of ITGA3-WT and ITGA3-MUT with miRNA-144-5p sequences; (b) the luciferase activity of TC cell line TPC-1 in different treatment groups; (c) mRNA expression of ITGA3 in TPC-1 and FTC-133 cells upon overexpression of miRNA-144-5p; (d) protein expression of ITGA3 in TC cell lines TPC-1 and FTC-133; ∗ denotes *p* < 0.05.

**Figure 5:** miRNA-144-5p regulates biological functions of TC by targeting ITGA3: (a, b) expression of ITGA3 mRNA and protein in different treatment groups; (c) proliferation of TPC-1 cells; (d) invasive potential of TPC-1 cells (100x); (e) migration potential of TPC-1 cells in different treatment groups (40x); (f) apoptosis level of TPC-1 cells; ∗ denotes *p* < 0.05.

**Table 1:** Primer sequences of qRT-PCR.

Gene	Sequence	
miRNA-144-5p	Forward primer	5′-GCGCGAATTCGAGATCTTAACAGACCCTAGCTC-3′
	Reverse primer	5′-GCGCGGATCCGTGCCCTGGCAGTCAGTAGG-3′

U6	Forward primer	5′-TGCGGGTGCTCGCTTCGGCAGC-3′
	Reverse primer	5′-CCAGTGCAGGGTCCGAGGT-3′

ITGA3	Forward primer	5′-TCAACCTGGATACCCGATTCC-3′
	Reverse primer	5′-GCTCTGTCTGCCGATGGAG-3′

GAPDH	Forward primer	5′-GTCTCCTCTGACTTCAACAGCG-3′
	Reverse primer	5′-ACCACCCTGTTGCTGTAGCCAA-3′

## Data Availability

The [DATA TYPE] data used to support the findings of this study are included within the article.
